# Exploring the Association between Glutathione Metabolism and Ferroptosis in Osteoblasts with Disuse Osteoporosis and the Key Genes Connecting them

**DOI:** 10.1155/2022/4914727

**Published:** 2022-05-12

**Authors:** Yuanlin Wang, Yiming Jia, Yujing Xu, Xingkun Liu, Zheng Wang, Yang Liu, Bing Li, Jun Liu

**Affiliations:** ^1^Department of Joints, Tianjin Hospital, Tianjin University, 300211, China; ^2^Clinical College of Orthopedics, Tianjin Medical University, Tianjin 300211, China; ^3^Department of Orthopedics, Chifeng Municipal Hospital, Chifeng 024000, China; ^4^Tianjin Key Laboratory on Technologies Enabling Development of Clinical Therapeutics and Diagnostics, School of Pharmacy, Tianjin Medical University, Tianjin 300070, China; ^5^School of Pharmacy, Tianjin Medical University, Tianjin 300211, China

## Abstract

Disused osteoporosis is a kind of osteoporosis, a common age-related disease. Neurological disorders are major risk factors for osteoporosis. Though there are many studies on disuse osteoporosis, the genetic mechanisms for the association between glutathione metabolism and ferroptosis in osteoblasts with disuse osteoporosis are still unclear. The purpose of this study is to explore the key genes and other related mechanism of ferroptosis and glutathione metabolism in osteoblast differentiation and disuse osteoporosis. By weighted gene coexpression network analysis (WGCNA), the process of osteoblast differentiation-related genes was studied in GSE30393. And the related functional pathways were found through the Kyoto Encyclopedia of Genes and Genomes (KEGG) pathway analysis. By combining GSE1367 and GSE100933 together, key genes which were separately bound up with glutathione metabolism and ferroptosis were located. The correlation of these key genes was analyzed by the Pearson correlation coefficient. GSTM1 targeted agonist glutathione (GSH) selected by connectivity map (CMap) analysis was used to interfere with the molding disused osteoporosis process in MC3T3-E1 cells. RT-PCR and intracellular reactive oxygen species (ROS) were performed. Two important pathways, glutathione metabolism and ferroptosis pathways, were found. GSTM1 and TFRC were thought as key genes in disuse osteoporosis osteoblasts with the two mechanisms. The two genes have a strong negative correlation. Our experiment results showed that the expression of TFRC was consistent with the negative correlation with the activation process of GSTM1. The strong relationship between the two genes was proved. Glutathione metabolism and ferroptosis are important in the normal differentiation of osteoblasts and the process of disuse osteoporosis. GSTM1 and TFRC were the key genes. The two genes interact with each other, which can be seen as a bridge between the two pathways. The two genes participate in the process of reducing ROS in disuse osteoporosis osteoblasts.

## 1. Introduction

Osteoporosis is one of the most common orthopedic diseases worldwide with age-related neurological disorders being its major risk factors [1]. Disuse osteoporosis belongs to secondary osteoporosis, which is mainly caused by the reduction of bone mechanical force. Spinal cord injury, hemiplegia, fracture, long-term bed rest, and space flight are the causes of disuse osteoporosis [2]. The specific mechanism of disuse osteoporosis is still unknown. The process of bone reconstruction is based on the dynamic balance of two main mechanisms: osteoclast-related bone absorption and osteoblast-related bone formation, accompanied by the effects of various stimuli in vivo and in vitro [3]. Mechanical stress stimulation plays an important role in maintaining the stability of bone metabolism and maintaining normal function [4]. Studies on osteoblast simulating microgravity have shown that 50% of cells will lose vitality after 6 weeks of culture [5]. These show that cell death occurring in osteoblasts is an important pathogenic mechanism of disuse osteoporosis.

Cell death is caused by a variety of mechanisms. Cell death modes include autophagy, pyroptosis, Wallerian degeneration, excitotoxicity, and ferroptosis [6–8]. Ferroptosis is a nonapoptotic cell death mode, which is significantly different from other programmed cell death [9]. The general process of ferroptosis can be decided two steps: (1) transferrin receptor 1 transports circulating iron to cells inside and (2) divalent iron ions are released to iron pool belonging to lysosomes [10]. The remote cause of this mechanism is usually due to the decline of glutathione synthesis and metabolism-related functions in cells, resulting in the excess of reactive oxygen species [11]. Many genes such as TFRC, P53, and GPX4 have been proved to be involved in the occurrence and development of ferroptosis [12–15]. As a mechanism related to intracellular metabolism, it has attracted extensive attention in a variety of immune diseases, malignant tumors, and osteoporosis [16, 17]. Ferroptosis not only occurs in osteoporosis but also affects the differentiation and development of bone marrow mesenchymal cells. The FA complementation group D2 (FANCD2) was proved to reduce the accumulation of iron and reactive oxygen species in the differentiation of bone marrow mesenchymal cells [18]. The increase of reactive oxygen species will cause the damage of mitochondria and other organelles and induce cell death through various signal pathways [19, 20]. Therefore, the process of ferroptosis can be indirectly regulated by regulating the reactive oxygen species. As an antioxidant, GSH can play a multiantagonistic role through glutathione peroxidase and glutathione S-transferases [21]. In an animal experiment related to parenteral nutrition, the addition of GSH was proved to significantly reduce the high oxidative stress of various organs caused by this nutrition [22]. Related to iron metabolism, the concentration of intracellular GSH gradually recovered and the expression of Ferroportin 1 (Fpn-1) was decreased by using 1 mM apocynin in SHSY5Y cells [23].

Some studies have also focused on the ferroptosis-related mechanism that occurred in osteoporosis. Type 2 diabetes is often accompanied by osteoporosis. High glucose could induce ferroptosis in MC3T3E1 osteoblasts by accumulating ROS and consuming intracellular glutathione. In type 2 diabetes osteoporosis rats' bone tissue, the level of glutathione peroxidase 4 seen as the ferroptosis marker was reduced, while it will recover to a relative normal level after deferoxamine intervention [24]. This study showed that the low expression of FtMt gene caused the subsequent accumulation of ferrous ions in hFOB1.19 cells through the ROS/PINK1/Parkin pathway. The sequent intervention on the upregulated expression of the gene showed the inhibition of ferroptosis and the recovery of osteogenic ability. These results show the potential value by targeting specific genes to regulate the ferroptosis process.

For disuse osteoporosis, there are few studies on ferroptosis and its related mechanisms and biomarkers. Recent studies found that the upregulation of DNA methylation-related DNMT1 and histone methylation-related EHMT2 genes would cause disused osteoporosis [25]. Past studies based on GSE100933 found that GSNAS1, SNHG12, and EPB41LA4A-AS1 can be seen as potential regulators in disuse osteoporosis [26]. GSH and ferroptosis have proved to be important in osteoblasts, while the key regulatory and potentially related genes are still unknown. Our study is aimed at exploring the relationship between the glutathione and iron metabolism pathway in normal osteoblasts and disuse osteoporosis osteoblasts.

In our study, we revealed the role of glutathione and iron metabolism pathway in osteoblast development. Then, we put two disuse osteoporosis datasets together and found that these two mechanisms played an important role in the occurrence of disused osteoporosis. The most important related regulatory genes, GSTM1 and TFRC, in the two mechanisms were discovered and that there was a strong correlation. In the cell experiment, GSH was added to detect its therapeutic effect and the relationship between two key genes.

## 2. Materials and Methods

### 2.1. Data Collection

Our overall workflow is shown in Figure 1. Three datasets were downloaded from the GEO database. The gene expression profiles GSE30393 related to MC3T3-E1 cells were acquired from the GEO database (http://www.ncbi.nlm.nih.gov/geo/), containing 12 samples which include different stages of osteoblast differentiation. GSE1367, related to 2T3 preosteoblasts, contains 3 static samples (control groups) and 3 microgravity samples. Another dataset, GSE100933, focuses on the bone marrow mesenchymal stem cells, which are the ancestors of preosteoblasts. This dataset contains four samples cultured in the standard medium onboard International Space Station (ISS) and other three samples cultured in the standard medium on ground. RStudio software based on R language was used to firstly deal with these data. The gene chip platform of the three datasets are separately GPL3108 (Duke University Microarray Facility Operon Mouse Oligo set, version 2.0), GPL6244 Illumina HumanWG-6 v3.0 expression, and GPL1219 Amersham Biosciences CodeLink UniSet Mouse I Bioarray. Ferroptosis-associated genes were downloaded from the FerrDb database (FerrDb (zhounan.org)). Glutathione metabolism pathway-related genes were downloaded from the DAVID database.

### 2.2. Dataset WGCNA Analysis

A coexpression network of GSE30393 was constructed by WGCNA R package about the days and differentiation stages of MC3T3-E1 cells. WGCNA R package is an open-source and widely used method in R language, which can be used to establish co expression network [27]. The gene expression data of 15301 genes in 12 samples of MC3T3-E1 cells at different differentiation stages and their corresponding differentiation characteristics (days and differentiation stage) were introduced into R software as basic information. Firstly, we cluster these samples through hclust methods to check the clustering degree and delete poor outliers. Subsequently, Pearson correlation analyses help us evaluate the relationship between gene pairs. A similarity matrix was constructed after that. After these preparation work, WGCNA started to be performed. The best soft threshold was selected to cluster the genes in the coexpression module to ensure that the scale independence is more than 0.85, and the average connectivity is close to 0. The dynamic tree cutting algorithm defines the module by cutting the component branches of the cluster tree and then assigns the module to different colors for visualization.

### 2.3. Screening of DEGs

limma R package was applied based on the classical Bayes *t*-test. In the GSE100933 dataset, ∣log_2_fold change (FC) | ≥1 and *P* < 0.01 were regarded as the thresholds for identifying significant DEGs. ∣log_2_fold change (FC) | ≥1 and P < 0.05 were the significant DEGs' criteria for GSE1367. Heatmap and volcano plots were utilized to visualize the expression levels of significant DEGs.

### 2.4. Functional Pathway Analysis of DEGs

DEGs from GSE10933 and genes belonging to key modules were matched with official gene symbol by using G: profile website (http://biit.cs.ut.ee/gprofiler/convert). KEGG pathway analysis of DEGs was performed with the help of the DAVID database and Cytoscape software. Bubble chart was obtained by R package “ggplot.” The Cluego plug-in unit in Cytoscape software was used to draw the relationship among the pathways.

### 2.5. Ferroptosis Related Genes and Protein-Protein Internet (PPI) Network Construction

Ferroptosis-related genes were obtained from the Ferrdb database. The Ferrdb database is the first in the world to summarize ferroptosis gene-related drivers, suppressors, and markers [28]. By using Venn-related website (Draw Venn diagrams, Result (ugent.be)), we can separately obtain the cross genes between ferroptosis-related genes and GSE1367 differential genes and GSE100933 differential genes. The String database was used to create a PPI network. The network was imported to Cytoscape software. Degree of these genes in network were calculated by plug-in cytoHubba (version 0.1) [29]. Degree ≥ 10 was thought as important genes. The common ferroptosis-related genes were selected by the Venn method. The common DEGs about the two mechanisms from GSE100933 and GSE1367 were selected by Venn methods.

### 2.6. Selection of Glutathione Metabolism Pathway-Related DEGs and PPI Network Construction

Glutathione metabolism pathway-related genes were obtained from the DAVID database (https://david.ncifcrf.gov/). Venn website (Draw Venn diagrams, Result (ugent.be)) was used to get the glutathione metabolism pathway-related GSE100933 DEGs. Then, we selected glutathione-related genes that appeared in both datasets. The network establishment is completed in the same way as the previous part.

### 2.7. Pearson Correlation Analysis

R package “ggpubr” was used to perform the Pearson correlation analysis between glutathione-related genes and ferroptosis-related genes [30]. ∣*R* | >0.8 was thought as strong correlation. And *P* value < 0.05 was considered statistically significant.

### 2.8. Targeted Compound Selection by CMap Analysis

We predicted the target compounds for GSTM1 and TFRC by using the CMap online tool (http://broadinstitute.org/cmap) [31]. This dataset tool could predict the agonists or antagonists that can work against a special gene.

### 2.9. PCR Validation and ROS Test

MC3T3E1 cells were obtained from CYAGEN Company. Cells were cultured in *α*-MEM medium and normal incubator environment. TRIzol reagent was used to extract total RNA, and then PrimeScript RT Reagent Kit helps inverse transcribe. Rotary Cell Culture System (RCCS) system from Synthecon Company which has been thought as effective in building disuse osteoporosis model was used [32]. MC3T3-E1 cells were firstly cultured on the surface of microcarrier. These cells attached to microcarriers were transferred in Rotary Cell Culture System (RCCS) system at a speed of 15 r/min for 2 days. We separately cultured these cells with normal MEM and added with 5 M glutathione DMEM. The replacement of normal MEM and 5 M GSH added medium was completed before molding. DCFH-DA probe (Sigma-Aldrich company), which could be detected by confocal microscopic, was used to observe the ROS in MC3T3-E1 cells. GraphPad Prism software and *t*-test were used to deal with corresponding data.

### 2.10. Statistical Methods

R package (version 3.6.2) and GraphPad prism software were used to perform statistical analysis. Multiple combinations of statistical analysis were utilized in analyzing DEGs. *t*-test was performed to process PCR data.

## 3. Results

### 3.1. Identification of Gene Coexpression Modules

Total 15301 genes were calculated in our study. Hierarchical clustering analysis was performed with R package “WGCNA.” To ensure a scale-free network, we chose the closest value, *β* = 9, as the soft threshold showed in Figure 2(a). The displayed dendrogram (Figure 2(b)) showed that the samples in this dataset have good clustering, and the meaningless grey modules do not occupy a large proportion. From Figure 2(c), we found that the *R*^2^ which could stand of the scale-free topology is 0.84. This meant that *β* = 9 was suitable for our analysis. Total 24 modules were screened (Figure 2(d)). Among them, black modules showed the strongest positive correlation with days and differentiation stage. So, we mainly focused on the genes in dark-orange modules. In black modules, we performed an analysis of the GS and MM. In our analysis (Figure 3(a)), the cor = 0.96, which revealed that there was a strong correlation between GS and MM showed a very significant correlation. At the same time, we chose MM > 0.8 and GS > 0.8 as the reference. Total 498 genes were selected. Subsequent functional analysis was also carried out on the basis of these 498 genes.

### 3.2. Screening of DEGs

According to our criteria, the DEGs of two datasets were shown in Figures 4(a) and 4(c). 60 DEGs were upregulated and 111 DEGs were downregulated in the GSE1367 dataset. 1226 DEGs were downregulated and 959 DEGs were upregulated in the GSE100933 dataset. The top 50 DEGs of two datasets were shown in Figures 4(b) and 4(d).

### 3.3. Functional Enrichment and Pathway Analysis of DEGs

The results of KEGG analysis about osteoblast differentiation-related genes showed that ribosome, lysosome, and glutathione metabolism and ferroptosis were the several main pathways (Figure 3(b)). For DEGs of GSE1367, we also found that glutathione metabolism was also one of the more important pathways (Figure 4(e)).

### 3.4. Ferroptosis- and Glutathione Metabolism-Related Genes

By using the Venn diagram to find common genes with ferroptosis (Figure 4(f)). Five DEGs from GSE1367 are listed in Table 1. Sixty-eight DEGs listed in Table 1 were chosen from GSE100933. And the common genes were TFRC and ENBB2. The PPI network of the 68 DEGs were built up (Figure 5(a)). And the hub genes were shown in Table 1 marked in red. Only TFRC belonged to the hub genes. DEGs selected from glutathione metabolism in GSE100933 formed a PPI network containing 4 genes (Figure 5(b)). The common genes of glutathione metabolism were GSTM1 (Figure 5(c)). This gene could also be located in the PPI network. So, GSTM1 was the key gene thought as glutathione metabolism related. TFRC was thought as the ferroptosis-related key gene.

### 3.5. The Correlation of Two Genes

The results of the Pearson correlation about two genes expression level were shown in Figure 5(d). In GSE30393, the *R* is -0.93 (*P* value = 1.6*e*-05). In GSE100933, the *R* is -0.82 (*P* value = 0.046). In GSE1367, the *R* is -0.92 (*P* value = 0.0097). The expression of the two genes has a strong negative correlation in both datasets, with significant statistical significance.

### 3.6. Predication of Targeted Compound

By inputting the gene symbol in the database, we got the targeted drug of the corresponding gene. Glutathione was screened as the only known agonist for GSTM1 (Table 2). However, we did not get the corresponding compound for the TFRC gene. Therefore, in the following cell experiments, we stimulated GSTM1 by adding glutathione to observe its effect on the disused osteoblast model and the subsequent expression of TFRC.

### 3.7. Validation of Glutathione- and Ferroptosis-Related Genes and ROS Tests

After adding glutathione, cells were cultured in the RCCS system at a speed of 15 r/min for 2 days. Through the confocal image (Figure 6(a)), we could find that a large number of ROS were produced after the modeling process of osteoblasts without glutathione. The modeling cells were shown in Figure 6(b). RT-PCR results (Figure 6(c)) showed that GSTM1 were upregulated after glutathione intervention. The expression of TFRC was downregulated. In the medium containing glutathione, the ROS produced by osteoblasts were significantly reduced.

## 4. Discussion

Intracellular ROS participate in the process of bone homeostasis by regulating the differentiation of osteoblasts and osteoclasts. Excessive production of ROS will prevent the differentiation and mineralization of osteoblasts [33]. Intracellular reduced glutathione can be involved in regulation of intracellular ROS. A study focusing on the low-molecular-weight protein tyrosine phosphatase (LME-PTP) revealed that the concentration of reduced glutathione increased with the increase of LME-PTP concentration in the first 21 days of osteoblast osteogenesis induction. This trend is consistent with the rapid proliferation and mineralization of osteoblasts [34]. In our study, the glutathione metabolism pathway-related genes were all upregulated. This is consistent with the increase of intracellular glutathione content. The function of glutathione metabolic pathway is closely related to the role of intracellular reducing glutathione. Iron metabolism also plays an important role in osteoblast differentiation. Iron ions are important for osteoblasts. It is widely recognized that iron overload or iron deficiency would inhibit the function of osteoblasts [35]. A study using iron chelator deferoxamine (DFO) showed that DFO reduced the expression of osteogenic gene and alkaline phosphatase while reducing the concentration of intracellular iron ion [36]. To some extent, these are closely related to our discovery that the ferroptosis pathway plays an important role in our research. This pathway involves the exchange of iron ions inside and outside cells and the metabolism of iron ions in cells. Osteoblasts can maintain the intracellular iron homeostasis during differentiation through this pathway.

Continuous energy supply is needed in all stages of osteoblast development and function. In the process of osteoblasts growth and differentiation, mitochondria produce reactive oxygen species through glycolysis and oxidative phosphorylation to meet the energy needs of osteoblasts [37]. Mitochondria with normal function can maintain the normal level of ROS in cells [38]. However, the imbalance of intracellular ROS occurs in various osteoblast-related diseases. Sun et al. [39] has witnessed that the accumulation of ROS in osteoblasts could significantly induce the apoptosis probability of MC3T3E1. Another study about the AlCl_3_-induced MC3T3-E1 cell osteoporosis found that ROS scavenger could alleviate the degree of mitophagy and apoptosis, restoring the normal function of cells [40]. Therefore, the role of ROS in the pathogenesis and treatment of osteoporosis should be widely concerned. A variety of genes involved in ROS have been proved to be closely related to the occurrence of osteoporosis. The absence of this GPX7 will lead to the decline of osteoblast osteogenic ability by the accumulation of ROS [41]. In osteoporosis related to type 2 diabetes mellitus, excessive iron accumulation in cells could induce ROS accumulation, which then caused the decline of osteoblast osteogenesis-related ability.

Our modeling process simulates the weightless environment and provides strong external stimulation for cells. After detecting the ROS level, we found that a lot of ROS were indeed produced after modeling. As the main enzymes for scavenging oxidative stress products, glutathione S-transferases which was encoded by GSTM1 can maintain normal bone mineral density by inhibiting the negative effect of oxidative stress. Glutathione S-transferases can use reduced glutathione to convert toxic substances in cells into nontoxic compounds, and glutathione can also be seen as an agonist of GSTM1 gene [42]. The expression of GSTM1 was upregulated after adding reduced glutathione. The addition of glutathione acts as an agonist for this gene. At the same time, we can see a significant decrease in ROS and an improvement in cell morphology. On the other side, ferroptosis related to mitochondrial ferritin (FtMt) can inhibit the ferroptosis process by reducing the accumulation of oxidative stress in hFOB1.19 cells [24]. In many kinds of diseases, such as sickle cell anemia and breast cancer, the deletion of GSTM1 had been witnessed to be closely related to the increase of intracellular iron concentration [43, 44]. In a study about bone mineral density (BMD) ofthe big joint, carriers with homozygous deletion of GSTM1 gene fragment were closely associated with lower BMD values at these joint sites [45].

In iron metabolism-related aspects, TFRC is an important participant in intracellular iron transport [46]. The protein that was transcribed and translated according to this gene can help transfer extracellular Fe^3+^ to intracellular [47]. In myeloma, the high expression of TFRC will induce the accumulation of iron concentration in cells. The accumulation could cause abnormal activation of osteoclasts and subsequent severe bone resorption [48]. TFRC mRNA overexpression influenced by ferric ammonium citrate in human osteoblast cells could decrease the osteogenesis-related mRNA expression of Runx2, alpha 1 collagen type I chain through the Hedgehog signaling pathway [49]. TFRC could induce the excessive intake of iron and then leads to excessive release of ROS through the NADPH oxidase 1 signal pathway [50]. Our bioinformatics analysis revealed that the two genes, GSTM1 and TFRC, were of significant correlation and might affect each other. In our study, GSTM1 was upregulated and TFRC was downregulated after cultivated in glutathione containing medium in RCCS system compared to MEM. Intracellular free reduced glutathione could combine with glutathione S-transferases and reduce the production of intracellular reactive oxygen species [51]. Our study shows that the addition of glutathione can activate GSTM1 in the process of modeling. At the same time, the expression of TFRC was downregulated, which might together play roles in reducing intracellular ROS. Of course, further research is needed in the future. And the two important pathways, ferroptosis and glutathione metabolism pathways, should also get more attention.

## 5. Conclusion

Our study firstly revealed that glutathione metabolism and ferroptosis pathway both play important roles in osteoblast differential process and disuse osteoporosis. Two key genes related to these two mechanisms, GSTM1 and TFRC, interact and affect each other. These can be regarded as the molecular biological basis for the communication between glutathione metabolism and ferroptosis. Glutathione, a GSTM1 agonist, was proved to effectively reduce the excessive ROS in osteoblasts. At the same time, the antagonistic relationship between GSTM1 gene and TFRC gene was also proved.

## Figures and Tables

**Figure 1:** Flow diagram shows the whole process of data collection, analysis, and cytological experiment.

**Figure 2:** (a) Network topology analysis of adjacency matrix under different soft thresholds. The soft thresholding power was marked clearly in red with a corresponding square value of correlation coefficient marked on the *y* axis. (b) Dendrogram on gene clustering and module allocation. (c) When scale-free topology is set to *β* = 9, the gene set with corresponding log10 and log10 *P* values. (d) Significant modules associated with the clinical traits (days and differential stages). Each cell in the chart shows a correlation with the trait. Red represents positive correlation, and green represents negative correlation.

**Figure 3:** (a) The relationship of GS and MM calculated in the DEGs from significant modules. Taking 0.8 as the boundary, the genes particularly related to the differentiation stage were segmented by lines. (b) KEGG pathway analysis of significant module genes. The size of the dot stands for the number of genes included in the pathway, and the color represents the *P* value.

**Figure 4:** (a, c) The volcano plot of DEGs in GSE1367 and GSE100933. The red nodes indicate the upregulated DEGs. The green nodes indicate the downregulated DEGs. (b, d) The heatmap of the top 50 DEGs. The expression levels of the top 50 DEGs in microgravity and healthy controls are shown contained in two datasets. Blue indicates low expression, and red indicates high expression. (e) KEGG pathway analysis of GSE100933 DEGs. Dots of different colors represent different pathways. The line represents connections between pathways. (f) Common genes of DEGs from two datasets related with ferroptosis. The green area represents GSE1367. The pink area represents GSE100933. The blue area represents ferroptosis-related genes.

**Figure 5:** (a) The PPI network of ferroptosis-related DEGs in GSE100933. The red represents upregulated, and orange represents downregulated. (b) The PPI network of ferroptosis-related DEGs in GSE100933. (c) Common genes of DEGs related with the glutathione metabolism pathway. The green area represents GSE1367. The pink area represents GSE100933. The blue area represents glutathione-related genes. (d) The Pearson correlation analysis of GSTM1 and TFRC in two disused datasets. The value of *X* axis represents the expression of TFRC. The value of *Y* axis represents the expression of GSTM1.

**Figure 6:** (a) Confocal photos of intracellular ROS detection. The green fluorescence is the intracellular oxidative stress product labeled by the probe. (b) Comparison of normal and modeled cells under optical microscope. (c) Relative mRNA expression in of TFRC and GSTM1 in the normal group (*n* = 5) and glutathione intervention group (*n* = 5). ^∗^*P* < 0.05, ^∗∗^*P* < 0.01.

**Table 1:** Ferroptosis- and glutathione metabolism-related genes.

Group	Ferroptosis	Glutathione metabolism
GSE100933	HSPB1, TRIB3, GOT1, LONP1, ACSL3, PLIN2, SCP2, RGS4, MT3, ACSF2, EIF2S1, PTGS2, GCH1, ENPP2, SLC7A11, TNFAIP3, GCLC, SLC2A1, SLC2A14, CXCL2, G6PD, MTDH, SLC3A2, RB1, LURAP1L, HILPDA, SAT1 PANX1, ATF3, CHMP5, SLC40A1, AKR1C2, SCD, CAPG, DUSP1, TGFBR1, NOX4, ACO1, GABARAPL1, CISD2, ATG13, GABPB1, TFRC, ARNTL, TXNIP, IL6, TUBE1, DDIT4, HERPUD1, SLC7A5, AIFM2, NQO1, DDIT3, HSPA5, WIPI1, RRM2, CAV1, CEBPG, MAPK3, ASNS, XBP1, SLC38A1, AKR1C3, JUN, SESN2, PGD, TP63	GCLM, GSTM4, TXNDC12, GCLC, GSTM1, ODC1, GSTM2, GSTA4 GSTT2, GSTK1, RRM2, GSTO1, PG,D
GSE1367	PLIN4, IDH1, ENPP2, TFRC, HNF4A	GSTM1, GSTT1, GGT5, IDH1
Common genes	TFRC, ENPP2	GSTM1

**Table 2:** The results of CMap analysis.

Compound	Molecular structure	Mechanism of action	Targeted genes
Glutathione		Antioxidant	GSTM1

## Data Availability

All data generated or analyzed during the present study are included in this published article. GSE30393 can be downloaded from: https://www.ncbi.nlm.nih.gov/geo/query/acc.cgi?acc=GSE30393. GSE1367 can be downloaded from: https://www.ncbi.nlm.nih.gov/geo/query/acc.cgi?acc=GSE1367. GSE100933 can be downloaded from: https://www.ncbi.nlm.nih.gov/geo/query/acc.cgi?acc=GSE100933.

## Abbreviations

WGCNA: Weighted gene coexpression network analysis
KEGG: Kyoto Encyclopedia of Genes and Genomes
CMap: Connectivity map
DEGs: Differential expression genes
PPI: Protein-protein interaction
GSH: Glutathione.

## References

[1] Anam A. K., Insogna K. (2021). Update on osteoporosis screening and management. *The Medical Clinics of North America*.

[2] Lindgren J. U., DeLuca H. F., Mazess R. B. (1984). Effects of 1, 25 (OH)2D3 on bone tissue in the rabbit: studies on fracture healing, disuse osteoporosis, and prednisone osteoporosis. *Calcified Tissue International*.

[3] Yang X. J., Wang F. Q., Lu C. B. (2020). Modulation of bone formation and resorption using a novel zoledronic acid loaded gelatin nanoparticles integrated porous titanium scaffold: an in vitro and in vivo study. *Biomedical Materials*.

[4] Song L. (2017). Calcium and bone metabolism indices. *Advances in Clinical Chemistry*.

[5] Camirand A., Goltzman D., Gupta A., Kaouass M., Panda D., Karaplis A. (2016). The role of parathyroid hormone-related protein (PTHrP) in osteoblast response to microgravity: mechanistic implications for osteoporosis development. *PLoS One*.

[6] Green J. L., Dos Santos W. F., Fontana A. C. K. (2021). Role of glutamate excitotoxicity and glutamate transporter EAAT2 in epilepsy: opportunities for novel therapeutics development. *Biochemical Pharmacology*.

[7] Llobet Rosell A., Neukomm L. J. (2019). Axon death signalling in Wallerian degeneration among species and in disease. *Open Biology*.

[8] Yao X., Li W., Fang D. (2021). Emerging roles of energy metabolism in ferroptosis regulation of tumor cells. *Advanced Science*.

[9] Ma H., Wang X., Zhang W. (2020). Melatonin suppresses ferroptosis induced by high glucose via activation of the Nrf2/HO-1 signaling pathway in type 2 diabetic osteoporosis. *Oxidative Medicine and Cellular Longevity*.

[10] Torii S., Shintoku R., Kubota C. (2016). An essential role for functional lysosomes in ferroptosis of cancer cells. *The Biochemical Journal*.

[11] Li J. Y., Yao Y. M., Tian Y. P. (2021). Ferroptosis: a trigger of proinflammatory state progression to immunogenicity in necroinflammatory disease. *Frontiers in Immunology*.

[12] Fang D., Wang Y., Zhang Z. (2021). Calorie restriction protects against contrast-induced nephropathy via SIRT1/GPX4 activation. *Oxidative Medicine and Cellular Longevity*.

[13] Luo Y., Gao X., Zou L., Lei M., Feng J., Hu Z. (2021). Bavachin induces ferroptosis through the STAT3/P53/SLC7A11 axis in osteosarcoma cells. *Oxidative Medicine and Cellular Longevity*.

[14] Yang J., Huang T., Petralia F. (2015). Synchronized age-related gene expression changes across multiple tissues in human and the link to complex diseases. *Scientific Reports*.

[15] Zhuang S., Ma Y., Zeng Y. (2021). METTL14 promotes doxorubicin-induced cardiomyocyte ferroptosis by regulating the KCNQ1OT1-miR-7-5p-TFRC axis. *Cell Biology and Toxicology*.

[16] Wang H., Lin D., Yu Q. (2021). A promising future of ferroptosis in tumor therapy. *Frontiers in Cell and Development Biology*.

[17] Xu W., Deng H., Hu S. (2021). Role of ferroptosis in lung diseases. *Journal of Inflammation Research*.

[18] Song X., Xie Y., Kang R. (2016). FANCD2 protects against bone marrow injury from ferroptosis. *Biochemical and Biophysical Research Communications*.

[19] Villalpando-Rodriguez G. E., Gibson S. B. (2021). Reactive oxygen species (ROS) regulates different types of cell death by acting as a rheostat. *Oxidative Medicine and Cellular Longevity*.

[20] Yang J., Huang T., Song W. M. (2016). Discover the network mechanisms underlying the connections between aging and age-related diseases. *Scientific Reports*.

[21] Nauser T., Koppenol W. H., Gebicki J. M. (2005). The kinetics of oxidation of GSH by protein radicals. *The Biochemical Journal*.

[22] Morin G., Guiraut C., Perez Marcogliese M., Mohamed I., Lavoie J. C. (2019). Glutathione supplementation of parenteral nutrition prevents oxidative stress and sustains protein synthesis in guinea pig model. *Nutrients*.

[23] Hou L., Huang R., Sun F., Zhang L., Wang Q. (2019). NADPH oxidase regulates paraquat and maneb-induced dopaminergic neurodegeneration through ferroptosis. *Toxicology*.

[24] Wang X., Ma H., Sun J. (2022). Mitochondrial ferritin deficiency promotes osteoblastic ferroptosis via mitophagy in type 2 diabetic osteoporosis. *Biological Trace Element Research*.

[25] Li B., Zhao J., Ma J. (2021). Cross-talk between histone and DNA methylation mediates bone loss in hind limb unloading. *Journal of Bone and Mineral Research*.

[26] Wei W. Z., Li B., Lin J. X. (2021). Analysis of long non-coding RNA expression profiles in disuse osteoporosis using microarray and bioinformatics. *Journal of Biological Regulators and Homeostatic Agents*.

[27] Langfelder P., Horvath S. (2008). WGCNA: an R package for weighted correlation network analysis. *BMC Bioinformatics*.

[28] Zhou N., Bao J. (2020). FerrDb: a manually curated resource for regulators and markers of ferroptosis and ferroptosis-disease associations. *Database: The Journal of Biological Databases and Curation*.

[29] Chin C. H., Chen S. H., Wu H. H., Ho C. W., Ko M. T., Lin C. Y. (2014). cytoHubba: identifying hub objects and sub-networks from complex interactome. *BMC Systems Biology*.

[30] Fang Y., Huang S., Han L., Wang S., Xiong B. (2021). Comprehensive analysis of peritoneal metastasis sequencing data to identify LINC00924 as a prognostic biomarker in gastric cancer. *Cancer Management and Research*.

[31] Lamb J., Crawford E. D., Peck D. (2006). The Connectivity Map: using gene-expression signatures to connect small molecules, genes, and disease. *Science*.

[32] Saxena R., Pan G., McDonald J. M. (2007). Osteoblast and osteoclast differentiation in modeled microgravity. *Annals of the New York Academy of Sciences*.

[33] Tao H., Ge G., Liang X. (2020). ROS signaling cascades: dual regulations for osteoclast and osteoblast. *Acta Biochimica et Biophysica Sinica Shanghai*.

[34] de Souza Malaspina T. S., Zambuzzi W. F., dos Santos C. X. (2009). A possible mechanism of low molecular weight protein tyrosine phosphatase (LMW-PTP) activity modulation by glutathione action during human osteoblast differentiation. *Archives of Oral Biology*.

[35] Ledesma-Colunga M. G., Weidner H., Vujic Spasic M., Hofbauer L. C., Baschant U., Rauner M. (2021). Shaping the bone through iron and iron-related proteins. *Seminars in Hematology*.

[36] Edwards D. F., Miller C. J., Quintana-Martinez A. (2021). Differential iron requirements for osteoblast and adipocyte differentiation. *JBMR Plus*.

[37] Karthik V., Guntur A. R. (2021). Energy metabolism of osteocytes. *Current Osteoporosis Reports*.

[38] Daneshgar N., Baguley A. W., Liang P. I. (2021). Metabolic derangement in polycystic kidney disease mouse models is ameliorated by mitochondrial-targeted antioxidants. *Communications biology*.

[39] Sun J. Y., Hou Y. J., Fu X. Y. (2018). Selenium-containing protein from selenium-enriched <i>Spirulina platensis</i> attenuates cisplatin-induced apoptosis in MC3T3-E1 mouse preosteoblast by inhibiting mitochondrial dysfunction and ROS-mediated oxidative damage. *Frontiers in Physiology*.

[40] Liu M., Wu X., Cui Y. (2021). Mitophagy and apoptosis mediated by ROS participate in AlCl_3_-induced MC3T3-E1 cell dysfunction. *Food and Chemical Toxicology*.

[41] Hu X., Li B., Wu F. (2021). GPX7 facilitates BMSCs osteoblastogenesis via ER stress and mTOR pathway. *Journal of Cellular and Molecular Medicine*.

[42] Dourado D. F., Fernandes P. A., Ramos M. J. (2010). Glutathione transferase classes alpha, pi, and mu: GSH activation mechanism. *The Journal of Physical Chemistry B*.

[43] Puri L., Flanagan J. M., Kang G. (2019). GSTM1 and liver iron content in children with sickle cell anemia and iron overload. *Journal of Clinical Medicine*.

[44] Sharma V., Kumar B., Saxena R. (2010). Glutathione S-transferase gene deletions and their effect on iron status in HbE/beta thalassemia patients. *Annals of Hematology*.

[45] Mlakar S. J., Osredkar J., Prezelj J., Marc J. (2011). Opposite effects of GSTM1– and GSTT1– gene deletion variants on bone mineral density. *Disease Markers*.

[46] Yao F., Cui X., Zhang Y. (2021). Iron regulatory protein 1 promotes ferroptosis by sustaining cellular iron homeostasis in melanoma. *Oncology Letters*.

[47] Leung K. (2004). (89) Zr-desferrioxamine B-transferrin. *Molecular Imaging and Contrast Agent Database (MICAD)*.

[48] Gu Z., Wang H., Xia J. (2015). Decreased ferroportin promotes myeloma cell growth and osteoclast differentiation. *Cancer Research*.

[49] Doyard M., Fatih N., Monnier A. (2012). Iron excess limits HHIPL-2 gene expression and decreases osteoblastic activity in human MG-63 cells. *Osteoporosis International*.

[50] Zhang L., Wang F., Li D., Yan Y., Wang H. (2021). Transferrin receptor-mediated reactive oxygen species promotes ferroptosis of KGN cells via regulating NADPH oxidase 1/PTEN induced kinase 1/acyl-CoA synthetase long chain family member 4 signaling. *Bioengineered*.

[51] Dafré A. L., Sies H., Akerboom T. (1996). Protein S-thiolation and regulation of microsomal glutathione transferase activity by the glutathione redox couple. *Archives of Biochemistry and Biophysics*.

